This article has been retracted.

# The Effect of CT Imaging Technology in the Diagnosis of Thoracic and Cardiac Surgery Diseases

**DOI:** 10.1155/2022/9385451

**Published:** 2022-08-24

**Authors:** Min Yang, Hongbo Qian, Dafa Zhang, Yingjing Gui

**Affiliations:** Cardiothoracic Surgery, The First Affiliated Hospital of Wannan Medical College (Yijishan Hospital), Wuhu, Anhui 241000, China

## Abstract

In order to increase doctors' cognition of the three-dimensional anatomical structure of cardiothoracic and cardiothoracic surgery and increase the diagnosis rate and cure rate of cardiothoracic surgery diseases, the authors propose a method of CT imaging technology for diagnosing cardiothoracic surgery diseases. Through the joint Hookwire positioning of 3D-CTBA, application in thoracoscopic segmentectomy and CT energy spectrum curve, retrospective analysis of diagnosis of intrathoracic lymph node metastasis in non-small-cell lung cancer, 3D-CTBA and CT-guided Hookwire localization, and preoperative CT-enhanced scanning were performed using two methods. The experimental results showed that the chest tube placement time, postoperative thoracic drainage volume, and postoperative hospital stay after the first operation all showed a good trend. The diagnostic sensitivity was 87.1%. The specificity was 92.6%. The correct index was 79.7%. The accuracy was 91.3%. The positive predictive value was 79.4%. And the negative predictive value was 95.7%. These data prove that CT imaging technology has high diagnostic value for thoracic and cardiac surgery diseases and can effectively help the formulation and implementation of thoracic and cardiac surgery diseases.

## 1. Introduction

Cardiothoracic surgery (Figure 1) is a highly specialized clinical discipline, involving many types of diseases, and new theories and technologies are updated rapidly; during the diagnosis and treatment process, doctors are required to be proficient in imaging and anatomy knowledge. Traditional (multimedia) clinical teaching methods are mainly based on lecture-style theoretical knowledge teaching and learning; although the teaching effect is relatively stable, it is difficult to stimulate students' enthusiasm and interest in learning. In addition, it lags behind the rapid development of diagnosis and treatment technologies (endoscopy, intervention, robot-assisted surgery, etc.), making it difficult for students to understand the three-dimensional anatomy of the cardiothoracic structure for clinical applications [1]. In recent years, CT imaging technology has been gradually applied in clinical teaching of orthopedics, neurosurgery, general surgery, and stomatology and achieved good results because of its immersion, interactivity, and conception effect. More importantly, the application of CT imaging-related technology in thoracic and cardiac surgery has achieved initial results, and many operations have achieved great success with the assistance of CT imaging technology [2]. Clinically, chest CT examination is the main examination method for the diagnosis of lung cancer; conventional CT can distinguish the size and texture of the tumor through iodine contrast, thereby judging the nature of the tumor. With the advancement of science and technology, the imaging resolution of CT has become higher and higher, and high-definition imaging has been achieved. Compared with other imaging methods, CT spectral imaging has higher spatial and temporal resolution. At the same time, it can avoid hardening artifacts and volume effects and can provide single-energy images and iodine-based images with the best contrast-to-noise ratio to enhance the display of iodine contrast agents, thereby avoiding omission and misdiagnosis of small lesions and improving the detection rate of small lesions and multiple lesions. The energy spectrum curve is the curve of the attenuation (CT value) of a substance or structure changing with the X-ray energy; from the energy spectrum curve, the average CT value and standard deviation of each energy point between 40 and 140 keV can be obtained [3]. The energy spectrum curve (CT value decay curve) is determined by the chemical molecular structure of the constituent substances; tissues with different chemical compositions have different CT value decay curves; the difference in CT value decay curves can be used to distinguish different chemical components in the human body. Therefore, in such a large environment, the authors propose to discuss the effect of CT imaging technology in diagnosing thoracic and cardiac surgery diseases. Objective analysis of CT imaging technology can reduce the time for finding and identifying lesions during surgery, minimize surgical damage, and preserve effective human tissue, so as to achieve anatomical, precise, and individualized treatment.

## 2. Literature Review

Visbal et al. found that 38.7% of severely calcified plaques on coronary CT scans were undiagnosed due to calcification artifacts [4, 5]. Coronary subtraction technology is to register the enhanced coronary CTA with the unenhanced calcification integral data, perform the overall deformable alignment based on the pixel grid model and the rigid alignment algorithm of local calcification, and then subtract it, which is a postprocessing technique. Calcified plaques and artifacts in the enhancement phase were eliminated by subtracting the data from two scans, followed by curved surface reconstruction for a more precise assessment of calcified stenosis. Liu et al. found that the 320-slice CT coronary subtraction technique can effectively overcome such calcification/sclerosis artifacts and improve the accuracy of diagnosis [6]. In order to obtain high-quality subtraction images, accurate alignment and registration of coronary CTA in the enhanced phase and calcium integral data in the plain scan phase are the key. Therefore, Fang et al. place the coronary unenhanced scan after the enhanced scan; the overall scanning time is shortened, and the patient can be scanned with one breath hold; however, the disadvantage of this method is that the residual iodine contrast agent cannot accurately calculate the calcification score during the plain scan [7]. Han et al. used the low-dose test method to shorten the two scan times within 20 s, and the patient completed one breath-holding scan. But the low-dose test method increases the amount of contrast injected. Therefore, the traditional “twice-holding” scanning method greatly reduces the requirement for long-term breath-holding scanning of patients and has the maximum application value. Due to individual differences, the quality of coronary subtraction images obtained from “two breath hold” scans is affected by many factors [8]. Cardillo and Emi found that the quality of CT pulmonary vein imaging depends on the best enhancement of the left atrium and proximal pulmonary vein, while the enhancement of the pulmonary artery is not obvious; that is, there is a significant difference in enhancement between the pulmonary vein and the pulmonary artery, which is helpful to distinguish the pulmonary artery from the pulmonary vein [9]. Because it is not easy to show the intersection of pulmonary artery branches and pulmonary veins at the hilar level, especially the main pulmonary artery and bilateral inferior pulmonary arteries, whether the pulmonary artery branches can be successfully removed during postprocessing, it is of great significance to determine whether there is variation in the bilateral upper pulmonary veins. The peak CT value of the pulmonary vein alone cannot guarantee the removal of the overlap of the pulmonary artery, which requires accurate estimation of the time when the contrast agent reaches the peak value and optimization of the injection plan; that is, the CT value of pulmonary artery and pulmonary vein and the difference between the two are used to quantitatively evaluate the effect of pulmonary vein imaging. Although there are different literatures at home and abroad concerning the enhancement scheme of MSCT pulmonary vein imaging, there is no unified opinion [10].

On the basis of current research, based on the application of 3D-CTBA combined with Hookwire localization in thoracoscopic segmentectomy and the CT energy spectrum curve, retrospective analysis of the diagnosis of intrathoracic lymph node metastases in non-small-cell lung cancer, by observing the surgical pathology and surgical process, the diagnostic value of CT imaging-related techniques was judged.

## 3. Methods

### 3.1. Scanning Trajectory Design

Common CT scan trajectories include circular trajectory, spiral trajectory, circular plus straight line, and double circle plus straight line. Since the circular trajectory does not meet the data completeness condition, it is not considered here [11]. Since the rotational motion of the object does not cause the overall movement of the two-axis electric object carrier, the motion range of the two-axis electric object carrier is completely determined by the translation stroke of the object. The following is an investigation of the translation travel required by the object in the latter three trajectories, and the trajectory with the shortest travel is selected as the scanning trajectory of the CT scanning system. It is assumed that the scanning radii of the above three trajectories are all *R*. The object support is a cylinder of radius *r* and height *H*. Let *μ* = *r*/*R*.

For a circle plus a straight line, point out that its translation stroke *T*_1_ (i.e., the length of the straight line) is at least

(1) $$\begin{array}{c} T_{1}=\frac{2H}{1-\mu }. \end{array}$$

That is, its translation stroke is more than twice the length of the phantom.

For the double circle plus straight line trajectory, point out that its translation stroke *T*_2_ (that is, the length of the straight line trajectory) is at least

(2) $$\begin{array}{c} T_{2}=H. \end{array}$$

That is, its translation stroke is equivalent to the length of the phantom.

For the helical trajectory, its translation travel *T*_3_ is at least

(3) $$\begin{array}{c} T_{3}=H+\left(1-\frac{\arccos\mu }{\pi }\right)\left(1+\mu \right)h, \end{array}$$

where *h* is the pitch of the helical trajectory, and its translation stroke is greater than the length of the phantom; the three trajectories are shown in Figures 2 and 3.

Comparing the three equations (1), (2), and (3), it can be seen that the translation stroke required by the double circle plus the linear trajectory is the smallest, and it is only related to the length of the phantom, and the width of the phantom and the parameters of the scanning trajectory are all related; it does not matter. In order to compare the three trajectories more intuitively, an example is given below. Assume that the scanning radius is *R* = 450 mm, the size of the phantom is *r* = 30 mm, and *H* = 100 mm. In order to make the rotation degree of the spiral track similar to the double circle plus straight line track, the pitch of the spiral track is selected as *h* = 50 mm. According to the above three formulas, there are *T*_1_ = 214.3 mm, *T*_2_ = 100.0 mm. It can also be seen that *T*_2_ is significantly smaller than *T*_1_. According to the above discussion, in the application of medical CT scanning, the double circle plus straight line trajectory is selected as the scanning trajectory [12].

### 3.2. Application of 3D-CTBA Combined with Hookwire Localization in Thoracoscopic Segmentectomy

#### 3.2.1. General Information

A retrospective analysis was performed on 48 patients with VATS segmentectomy in the Department of Thoracic and Cardiovascular Surgery of a hospital in a city, including 22 males and 26 females, with an average age of 59.75 ± 9.46 years. All patients had no obvious symptoms and signs such as cough, sputum, and blood in sputum, and the presence of pulmonary nodules was confirmed by chest thin-section CT. There were 56 small pulmonary nodules in 48 patients, including 48 GGN, 6 solid nodules, and 2 partially solid nodules. Among them, 2 nodules were <8 mm in diameter, 24 were 8-10 mm in diameter, and 30 were 11-20 mm in diameter, with an average diameter of 12.08 ± 3.48 mm. All patients underwent three-dimensional reconstruction with Mimics Medical 20.0 software before operation and were positioned with Hookwire under CT guidance and then sent to the operating room for surgical treatment, with preoperative routine improvement of three routines, chest enhanced CT, head MRA, abdominal color Doppler ultrasound, bone ECT scan, and cardiopulmonary function examinations [13].

1. *Inclusion Criteria*. (1) Unable to tolerate lobectomy; (2) nodules located in 1/3 around the lung field, with a diameter of ≤2 cm; (3) if it is a malignant tumor, it should be non-small-cell carcinoma, and the tumor stage is T1N0M0; (4) CT shows that the ground glass component is ≥50%, and the doubling time is ≥400 days; (5) lymph node biopsy excludes distant metastasis; (6) no previous thoracotomy or previous diseases that cause pleural adhesions; (7) Indications for VATS surgery; and (8) voluntary participation in this study and signed informed consent [14].
2. *Exclusion Criteria*. (1) Patients with severe heart and lung dysfunction, unable to tolerate surgery, with abnormal coagulation function, and unable to tolerate one-lung ventilation tuberculosis; (2) mental disorders; (3) refusal of the study or resistance of the operation.

#### 3.2.2. Specific Method

1. *3D-CTBA and CT-Guided Hookwire Localization*. All patients underwent chest enhanced CT examination before surgery, and the imaging data were imported into Mimics Medical 20.0 software in DICOM format, and the surgeon and an assistant jointly constructed a three-dimensional reconstructed image [15]. Identify the lung segment where the nodule is located, analyze the course of the arterial (venous) artery and bronchi and the anatomical structure relationship of the target segment, observe whether there is variation, and mark it with different colors. The surgical team discussed the surgical plan, planned the best surgical path, and performed simulated surgery.
2. *Preoperative Preparation*. All patients were intramuscularly injected with pethidine 50 mg before positioning, and appropriate body positions were taken according to the position of the nodule after three-dimensional reconstruction and the surgical approach, and the patients were instructed to keep a relatively static state and a relatively stable breathing range as much as possible [16]. CT scan is performed to display the location of the target lesion. The radiologist and the surgeon will negotiate to determine the optimal intercostal and angle of needle insertion, measure the distance between the lesion and the chest wall, and determine the depth of needle insertion. Then use the CT laser positioning line to establish the body surface positioning mark, and place a metal positioning mark ruler at the body surface positioning line. Perform routine disinfection, drape, local infiltration anesthesia, and insertion into the parietal pleura according to the planned puncture route. CT scan was performed again to determine whether the direction of the puncture needle was facing the lesion, and if there was a deviation, a small angle was adjusted. Then, insert the needle into the lesion, withdraw the needle core, rapidly expand and release the Hookwire positioning needle, repeat the CT scan, and confirm that the positioning needle is located in the lesion or not more than 5 mm away from the lesion. The skin was flushed, and the metal wire was cut, bandaged with gauze and fixed with tape, and sent to the operating room for surgical treatment [17]. According to imaging manifestations, clinical symptoms, and intraoperative exploration, determine whether the patient has pneumothorax or hemothorax due to localization, and record the time of localization.
3. *Surgical Method*. After the double-lumen endotracheal intubation was stabilized under general anesthesia, the patient was placed in a lateral decubitus position, the surgical field was routinely disinfected, and a sterile drape was laid. Usually, a 1.5 cm incision is made at the posterior axillary line of the seventh intercostal space, the thoracic cavity is separated layer by layer, one-lung ventilation is performed, and a 1.2 cm Trocar is inserted into the thoracoscope, exploring whether there is pleural effusion and adhesion and observing the development of lung surface and hilar lymph nodes. Under the guidance of a thoracoscope, make a 5.0 cm incision on the anterior axillary line of the fourth intercostal space, introduce instruments, find the positioning needle, and determine the target segment based on preoperative 3D-CTBA images. According to the surgical path planned before operation, dissect the target bronchus, arteries, and veins and try to dissociate along the vascular sheath to the distal end during the dissection, carefully identify and operate with caution, preserve the intersegmental veins, reveal the plane of the lung segment by the inflation and collapse method and mark for separation, use a straight cut suture to completely resect the lung segment, and send for rapid pathological examination. If the pathological result is a benign nodule, atypical adenomatous hyperplasia, adenocarcinoma in situ, or minimally invasive adenocarcinoma, the operation is over. If the pathological result is invasive adenocarcinoma, routinely sample and dissect N1 and N2 lymph nodes, and send for rapid pathological examination; lobectomy+systemic lymph node dissection was performed instead (lymph node metastasis was excluded in this study).
4. *Observation Indicators*. According to imaging manifestations, clinical symptoms, and intraoperative exploration, determine whether the patient has pneumothorax or hemothorax due to positioning, and record the positioning time. The operation time and intraoperative blood loss were statistically analyzed according to the anesthesia records, and the postoperative chest tube intubation time, postoperative chest drainage volume, and postoperative hospital stay were statistically analyzed according to the postoperative nursing records; postoperative complications were recorded according to patient symptoms and imaging data, and pathological data were recorded according to intraoperative rapid pathology and postoperative routine pathology [18].

#### 3.2.3. Statistical Analysis

All data were entered and analyzed using SPSS 22.0, and the data in this study were expressed as the mean ± standard deviation.

#### 3.2.4. The Diagnosis of Intrathoracic Lymph Node Metastasis in Non-Small-Cell Lung Cancer by CT Energy Spectrum Curve

*(1) General Information*. 53 patients with non-small-cell lung cancer who were diagnosed and treated in a hospital in a certain year and month were selected; all patients underwent radical surgery for lung cancer and were confirmed by pathology. Among them, 27 were male and 26 were female; 17 were squamous cell carcinoma, 36 were adenocarcinoma, 41 were peripheral lung cancer, and 12 were central lung cancer. The general information of the patients is shown in Tables 1 and 2.

*(2) Specific Methods*. All patients underwent enhanced CT scans before surgery. Spectral imaging was performed using a GE HealthCare discovery CT 750 HD; the tube voltage was switched instantaneously between 80 kVp and 140 kVp, the tube current was 600 mA, the layer thickness was 5.0 mm, the interval was 5.0 mm, the matrix was 512 × 512, the pitch was 1.375 : 1, and the rotational speed was 0.6 s/cycle or 0.8 s/cycle. The enhanced scan was performed using a German Orrich double-barrel high-pressure syringe, and 370 mgI/ml of Univitamin was injected through the median cubital vein at a dose of 70 ml, followed by 30 ml of normal saline at a rate of 4.0 ml/s, the arterial phase, and the venous phase. The delay period starts scanning at 25, 55, and 140 s, respectively. The primary lesions and CT-visible lymph nodes were analyzed by energy spectrum. The original data was reconstructed into an image set with a slice thickness of 0.625 mm under the single-energy reconstruction algorithm and transferred to the postprocessing workstation GEAw 4.5 (GE HealthCare, USA); all data were analyzed and processed using GSIViewer software. Select the homogeneous part of the lesion as the region of interest; try to avoid necrotic tissue, cavities, calcifications and blood vessels, etc.; measure the energy spectrum curve of the region of interest and calculate the slope of the curve; according to the slope of the energy spectrum curve between 40 and 140 keV, diagnosis was made and divided into the metastatic and nonmetastatic groups [19].

*(3) Related Standards*. *Diagnostic criteria*: when the difference between the energy spectrum slopes of the primary tumor and the lymph node is less than 0.2, the two curves are considered to be consistent [20]. If the primary tumor is homologous to the lymph node, the lymph node is considered a metastatic lymph node; otherwise, there is no metastasis. *Gold standard*: the gold standard is surgical dissection and marking of intrathoracic lymph nodes and pathological diagnosis to determine whether metastatic lymph nodes are present. Create a matching four-table, using pathological diagnosis as the gold standard, the diagnostic results of spectral CT were evaluated.

*(4) Evaluation Indicators*. Calculate accuracy, sensitivity, specificity, misdiagnosis rate, missed diagnosis rate, positive predictive value, negative predictive value, and correct index, in order to evaluate the diagnostic value of the CT energy spectrum curve for intrathoracic lymph node metastasis of non-small-cell carcinoma.

## 4. Results and Discussion

Hookwire positioning under CT guidance was successfully performed, and the average positioning time was 19.71 ± 3.94 min; intraoperative exploration clearly showed the complete Hookwire, no positioning needle displacement and falling off, and no residue. Combined with the patient's imaging data, symptoms, and lung surface exploration, 5 cases of pneumothorax occurred, but no hemothorax; after timely symptomatic treatment such as oxygen inhalation and puncture, the implementation of VATS was not affected. All patients successfully completed VATS according to the preoperative plan; there was no conversion to thoracotomy. The intraoperative anatomy was basically the same as the preoperative 3D reconstruction image, the nodule was located accurately, and the resection margin met the oncological requirements; the specific lung segment statistics are shown in Figure 4. The average operation time was 109.67 ± 17.21 min, intraoperative blood loss was 65.42 ± 21.62 ml, postoperative chest tube placement time was 4.13 ± 1.26 d, postoperative chest drainage volume was 548.33 ± 228.78 ml, and the postoperative hospital stay was 6.25 ± 1.48 d. Postoperative complications occurred in 6 cases, including 1 case of chylothorax, 1 case of pulmonary infection, 2 cases of arrhythmia, and 2 cases of pulmonary air leakage; all patients were discharged after active symptomatic treatment, and there were no deaths [21].

*Pathological data*: there were 2 cases of inflammatory granuloma, 2 cases of bronchiolar adenoma, and 3 cases of inflammatory nodules. There were 1 case of squamous cell carcinoma, 2 cases of atypical adenomatous hyperplasia, 3 cases of adenocarcinoma in situ, 14 cases of invasive adenocarcinoma, and 29 cases of minimally invasive adenocarcinoma, all without lymph node metastasis.

The patients in this group underwent radical surgery for lung cancer from Table 3, the pathological diagnosis was non-small-cell lung cancer, and 126 groups of lymph nodes were analyzed by the energy spectrum curve. Among them, GSI diagnosed metastatic lymph nodes in 31 groups (slope 1.19 ± 0.14) and nonmetastatic lymph nodes in 95 groups (slope 1.87 ± 0.23). There were 115 groups that were consistent with the pathological results and 11 groups that were not. Among them, the pathological results were metastatic lymph nodes, while the energy spectrum analysis showed that there were 4 groups of nonmetastatic lymph nodes, with a missed diagnosis rate of 12.9% (among them, R4 lymph node group 1, L10 lymph node group 1, R11 lymph node group 1, and L11 lymph node group 1). The pathological results were nonmetastatic lymph nodes, while the energy spectrum analysis showed that there were 7 groups of metastatic lymph nodes, with a misdiagnosis rate of 7.4% (among them, group 7 lymph node group 3, R10 lymph node group 2, R4 lymph node group 1, and L4 lymph node group 1). The sensitivity was 87.1%. The specificity was 92.6%. The correct index was 79.7%.. The accuracy was 91.3%. The positive predictive value was 79.4%. And the negative predictive value was 95.7%.

Clinically, chest CT examination is the main examination method for the diagnosis of lung cancer; conventional CT can distinguish the size and texture of the tumor through iodine contrast, thereby judging the nature of the tumor [22]. With the advancement of science and technology, the imaging resolution of CT is getting higher and higher, and high-definition imaging has been realized. Compared with other imaging methods, CT spectral imaging has higher spatial and temporal resolution. At the same time, it can also avoid hardening artifacts and volume effects and can provide single-energy images and iodine-based images with the best contrast-to-noise ratio to enhance the display of iodine contrast agents, thereby avoiding omission and misdiagnosis of small lesions and improving small lesions and multiple lesions and detection rate [23]. Spectral CT uses the instantaneous switching of high and low dual energy (80 kVp and 140 kVp) of a single tube (<0.5 ms energy time resolution) to generate dual energy data, realize data space energy spectrum analysis, and provide material density images and single-energy image; material separation can be achieved, and the characteristic energy spectrum curve of material can be obtained [24]. The energy spectrum curve is the curve of the attenuation (CT value) of a substance or structure with the X-ray energy. From the energy spectrum curve, the average CT value and standard deviation of each energy point between 40 and 140 keV can be obtained. The energy spectrum curve (CT value attenuation curve) is determined by the chemical molecular structure of the constituent substances, different chemically composed tissues have different CT value attenuation curves, and the difference in the CT value attenuation curve can be used to distinguish different chemical components in the human body. Substances with different components have different slopes of decay curves, but the slopes are similar, indicating that there is homology between the two. By comparing the energy spectrum slopes of mediastinal and intrapulmonary lymph nodes with the primary lesion, it was judged whether it was a metastatic lymph node.

## 5. Conclusion

Through the joint Hookwire positioning of 3D-CTBA, application in thoracoscopic segmentectomy and CT energy spectrum curve, a retrospective analysis of the diagnosis of intrathoracic lymph node metastases in non-small-cell lung cancer, through 3D-CTBA and CT-guided Hookwire localization, and preoperative CT enhanced scanning energy spectrum imaging, the time of chest tube placement, postoperative thoracic drainage, and postoperative hospital stay were observed after the two operations, in order to prove that CT imaging technology has a beneficial effect on the diagnosis of thoracic and cardiac surgery, which is embodied in the higher spatial and temporal resolution of CT imaging and is more accurate.

## Figures and Tables

**Figure 1:** Principle of CT imaging.

**Figure 2:** Circle plus straight line trajectory.

**Figure 3:** Double circle plus straight line trajectory.

**Figure 4:** Intraoperative anatomy and preoperative 3D reconstructed images.

**Table 1:** General information/case of 53 patients with non-small-cell lung cancer.

Project	Number of cases	Project	Number of cases	Project	Number of cases
Gender		Tumor location		TNM staging	
Male	27	Upper right lobe	14	IA	7
Female	26	Right middle lobe	6	IB	10
Age		Lower right lobe	12	IA	11
<50	5	Upper left lobe	9	IB	13
50-60	13	Lower left lobe	12	IMA	7
60-70	28			IMB	5
>70	7			V	0

**Table 2:** Types/cases of 53 patients with non-small-cell lung cancer.

Project	Number of cases
Types of non-small-cell lung cancer	13
Squamous cell carcinoma	17
Adenocarcinoma	36

**Table 3:** Parts of lung segments resected in 48 patients with thoracoscopic segmentectomy (cases).

Lung segment	Right lung	Left lung
S1	4	1
S2	5	0
S3	8	0
S1 + 2	0	5
S1 + 2 + 3	0	7
S4 + 5	0	2
S6	5	7
S7 + 8	1	1
S8	1	1
S9	I	0
S10	2	1
S9 + 10	1	0

## Data Availability

The data used to support the findings of this study are available from the corresponding author upon request.
